# High Glucose Induces Bone Marrow-Derived Mesenchymal Stem Cell Senescence by Upregulating Autophagy

**DOI:** 10.1371/journal.pone.0126537

**Published:** 2015-05-11

**Authors:** Tzu-Ching Chang, Min-Fen Hsu, Kenneth K. Wu

**Affiliations:** 1 Metabolomic Medicine Research Center, China Medical University Hospital, Taichung, Taiwan; 2 Graduate Institute of Clinical Medical Science, China Medical University, Taichung, Taiwan; 3 Graduate Institute of Basic Medicine, China Medical University, Taichung, Taiwan; 4 National Health Research Institutes, Zhunan, Taiwan; University-Hospital of Parma, ITALY

## Abstract

Hyperglycemia was reported to cause bone marrow hematopoietic niche dysfunction, and high glucose (HG) in the cultured medium induces MSC senescence. The underlying mechanism is unclear. Here, we investigated the role of HG-induced autophagy in bone-marrow-derived mesenchymal stem cell (BMSC) senescence. HG (25 mM) increased expression of Beclin-1, Atg 5, 7 and 12, generation of LC3-II and autophagosome formation which was correlated with development of cell senescence. Pretreatment of HG-MSC with 3-methyladenine (3-MA) prevented senescence but increased apoptosis. N-acetylcysteine (NAC) was effective in abrogating HG-induced autophagy accompanied by prevention of senescence. Diphenyleneiodonium (DPI), an inhibitor of NADPH oxidase, blocked autophagy and senescence in a manner comparable to NAC. 3-MA, NAC and DPI inhibited HG-induced interleukin-6 production in BMSCs. These results suggest that hyperglycemia induces MSC senescence and local inflammation via a novel oxidant-mediated autophagy which contributes to bone marrow niche dysfunction and hematopoietic impairment.

## Introduction

Hyperglycemia due to diabetes mellitus and metabolic syndrome has emerged as a major problem that threatens health and causes vascular and organ dysfunction. Recent reports indicate that hyperglycemia impairs bone marrow hematopoietic function and alters hematopoietic niche [1]. Diabetes was reported to alter chemokine expression on bone marrow multipotent mesenchymal stromal cells (also known as mesenchymal stem cells or MSCs) [2]. Bone Marrow-derived MSCs (BMSC) cultured in medium containing high glucose (HG) concentrations were reported to exhibit premature senescence, genomic instability and telomere changes [3–5]. The mechanism by which HG induces BMSC senescence is unclear. We postulated that HG suppresses BMSC autophagy thereby accelerating their senescence. Surprisingly, the results reveal that HG upregulated expression of Beclin-1, Atg 5, 7 and 12 and increased LC3-II generation and autophagosome formation, which were correlated with senescent changes in BMSC. Inhibition of autophagy with 3-methyladenine (3-MA) prevented senescence. Furthermore, treatment of BMSC with an antioxidant, N-acetylcysteine (NAC) or an NADPH oxidase inhibitor, diphenyleneiodonium chloride (DPI), abrogated HG-induced autophagy upregulation, premature senescence and interleukin-6 (IL-6) production.

## Methods

### Cell culture

Human BMSCs were routinely cultured in Dulbecco’s modified Eagle’s medium (DMEM) containing low-glucose (1.0 g/ L, 5.5mM) and supplemented with 10% fetal bovine serum (Hyclone), 100 U/ml penicillin and 100 μg/ml streptomycin at 37°C in a humidified 5% CO_2_ atmosphere. For this study, cells were washed and divided into two groups: one group was cultured in low-glucose (LG) and the other in high-glucose (HG) (4.5 g/L, 25 mM). Rapamycin, 3-methyladenine (3-MA), N-acetyl-L-cysteine (NAC) and diphenyleneiodonium chloride (DPI) were purchased from Sigma-Aldrich.

### Population doubling and BrdU analysis

For population doubling (PD) analysis, 1.5x10^5^ BMSCs were seeded and subcultured weekly. Cell number was determined by trypan blue assay. Cells were trypsinized, resuspended in medium, and viable cells were counted by using a hemocytometer. Cumulative PD at each subcultivation was calculated from the cell count by using the equation: Nh/Ni = 2^x^ where Ni = inoculum number, Nh = cell harvest number, and X = population doublings [6]. Cell proliferation was analyzed with bromodeoxyuridine (BrdU) assay kit (Chemicon). In brief, cells were incubated with 20 μM of BrdU before cells were harvested. Cells were treated with HCS fixation solution (1X) for 30 min. at RT. Mouse anti-BrdU antibody was added to cells for 1 hr. at RT. Cells were washed and goat anti-mouse IgG was added for 1 hr. at RT. Cells were washed and incubated with TMB peroxidase substrate for 30 min. The reaction was stopped and analyzed with a multimode microplate reader at 450 nm.

### Senescence associated β-galactosidase staining

Expression of pH-dependent senescence associated β-galactosidase (SA-β-gal) in BMSCs was analyzed using a SA-β-gal staining kit (Cell Signaling Technology). Briefly, BMSCs were washed and incubated in a fixative solution. β-Gal staining solution (final concentration 1mg/ mL of X-gal in DMF) was added and incubated at 37°C overnight. SA-β-gal stained cells were examined under light microscopy and quantified.

### Western blot analysis

Western blotting was performed as previously described [7]. Rabbit polyclonal antibodies against Beclin-1, LC3, cleaved caspase-3 and Poly-ADP-ribose polymerase (PARP) were from Cell Signaling. Mouse monoclonal antibodies against B-actin were from Sigma. Rabbit polyclonal and mouse monoclonal antibodies against p16 and p21 were from GeneTex Company.

### Quantitative real-time PCR (qPCR) analysis

Total RNA was isolated using TRIzol reagent (Invitrogen, Paisely, Scotland) according to the manufacturer’s instructions. RNA concentration was quantified with a NanoDrop ND-1000 Spectrophotometer (Nanodrop Technologies) and RNA quality was checked with the ratio of 260/280. Quantification of mRNA expression for candidate genes was performed by qPCR using ABI One-step Detection System Instrument (Applied Biosystems). Total RNA was reverse-transcribed by using high capacity cDNA reverse transcription kit (Invitrogen). qPCR reactions were performed with the power SYBR Green PCR Master mix (Roche) in a MicroAmp optical 96-well reaction plate according to the manufacturer’s instructions. Relative gene expression levels were normalized to GAPDH expression. The primer sequences of each genes for qPCR were as follows. Atg 5: forward primer (F), 5’-CCCTCCAGAAGAAAATGGAT-3’; and reverse primer (R), 5’-ATAGCTCAGATGCTCGCTCA-3’; Beclin-1: F, 5’-ACCGTGTCACCATCCAGGAA-3’; and R, 5’-GAAGCTGTTGGCACTTTCTGT-3’; Atg 7: F, 5’-TGTCAGCCTGGCATTTGATAA-3’; and R, 5’-TCACTCATGTCCCAGATCTCA-3’; Atg 12: F, 5’-TTCGGTTGCAGTTTCGCC-3’; and R, 5’-CCATGCCTGTGATTTGCAGTA-3’; GADPH: F, 5’-GAAATCCCATCACCATCTTCCAGG-3’; and R, 5’-GAGCCCCAGCCTTCTCCATG-3’.

### Detection of autophagosomes

Autophagosomes were detected with an autofluorescent compound monodansylcadaverine (MDC), using a Cell Meter Autophagy kit (AAT Bioquest, Inc.). Briefly, BMSCs were seeded on glass coverslips in a 24-wells plate at a density of 3 x 10^4^/well. After incubation, BMSCs were stained with 1 x MDC solution and incubated at 37°C for 1 hour. Cells were washed three times and examined under a confocal microscope (Ex = 330 nm).

### TUNEL assay

Terminal deoxynucleotidyl transferase-dUTP nick and labeling (TUNEL) assay for apoptosis was performed using the Click-iT TUNEL Alexa Flour 488 Assay kit (Molecular Probes, Inc) according to the manufacturer’s instructions. Briefly, cells were seeded in a 96-well microplate. After treatment, cells were fixed with 4% paraformaldehyde and then permeabilized with 0.2% Triton X-100. Transferase incorporation of EdUTP into dsDNA breaks was carried out in optimal reaction buffer at 37°C for 1h. Fluorescent detection of EdUTP was performed by click chemistry reaction for 30min and recorded with the excitation at 495nm and emission at 519nm.

### Analysis of reactive oxygen species (ROS)

BM-MSCs were incubated in a medium containing 10μM DCFH-DA at 37°C in the dark for 20min. The fluorescence intensity was detected by a flow cytometer (BD Biosciences) with the excitation at 488nm and emission at 535nm.

### Measurement of IL-6

IL-6 in the medium of cultured BMSCs was determined with an ELISA kit (Abcam) according to the manufacturer’s instructions. Briefly, a monoclonal antibody specific for IL-6 was coated onto the wells of microtiter plates. Samples and IL-6 standards were pipetted into wells. After incubation and washing, biotinylated monoclonal antibody specific for IL-6 was added, followed by streptavidin-HRP and TMB substrate. A standard curve was constructed and IL-6 concentrations in the samples were measured.

### Statistical analysis

Differences between groups were analyzed by Student *t* test. A *p* value of less than 0.05 was considered statistically significant.

## Results

### High glucose (HG) induces BMSC senescence

BMSCs cultured in HG exhibited a time-dependent reduction in cumulative PD (Fig 1A) and BrdU incorporation (Fig 1B). Cells cultured in HG for 2 weeks already show increased p16 and p21 (Fig 1C). HG also induced a time-dependent increase in SA-βgal positive cells (Fig 1D). Glucose at concentrations lower than 5.5. mM such as 2.75 mM did not affect BMSC cell morphology or numbers (Fig 1E). By contrast, glucose at 25 mM induced morphological changes consistent with senescence (Fig 1E). Taken together, these results indicate that compared to LG, chronic exposure to HG leads to progressive development of cellular senescence.

**Fig 1:** HG induces BMSCs senescence. **(A)** HG reduces cumulative PD. Cumulative PD was determined in BMSCs incubated in HG or LG for various time periods up to 28 days. HG-treated cells exhibit a time-dependent reduction of cumulative PD. **(B)** HG reduces BrdU incorporation. BrdU incorporation was measured in BMSCs incubated with HG or LG for various time periods. HG induced a progressive reduction of BrdU incorporation. **(C)** HG increases the expression of p16 and p21 proteins. BMSCs were incubated in medium containing HG or LG for 2 weeks and p16 and p21 proteins were analyzed by Western blotting. The left panel shows representative blots while the right panel, the densitometry of the blots. Error bars denote means ± SEM (n = 3). **(D)** HG induces SA-β-Gal. BMSCs cultured in HG or LG for 7 to 28 days were stained for SA-β-Gal and examined under light microscopy. Cells with positive SA-β-Gal staining were counted. HG increased SA-β-Gal in a time-dependent manner whereas LG did not have a significant effect on SA-β-Gal. **(E)** HG alters BMSC morphology. BMSCs were washed and incubated in medium containing various concentrations of glucose for 28 days: 2.75 and 5.5 mM are considered to be LG and 25 mM, HG. Cells became flat and rounded when cultured in HG. Error bars denote mean ± SEM (n = 3).

### HG-induced senescence is mediated by autophagy

HG increased BMSC Beclin-1 protein and LC3-II (Fig 2A), as well as Beclin-1, Atg 5, 7, and 12 mRNA (Fig 2B). To ensure that HG induces autophagosome formation, we analyzed autophagosomes by MDC staining. Cells cultured in LG exhibited a low level of autophagosomes which was greatly increased by HG (Fig 2C). Rapamycin increased while 3-MA blocked HG-induced autophagosome staining (Fig 2C). These results indicate that HG induces BMSC autophagy.

**Fig 2:** HG-induced autophagy related gene expression and autophagosome formation. BMSCs were incubated in medium containing LG (5.5 mM) or HG (25 mM) and autophagy was analyzed at 2 weeks. **(A)** Beclin-1 and LC3 were analyzed by Western blotting. Left panel shows a representative Western blot and right panel, densitometry of Western blots. The error bars denote mean ± SEM (n = 3). **(B)** Beclin-1 and Atg 5, 7 and 12 transcripts were measured by real time qPCR. Error bars denote mean ± SEM (n = 3). **(C)** BMSCs in LG or HG were treated with MDC and examined under fluorescent microscopy. RA and 3MA denote rapamycin (5 μM) and 3-methlyadenine (10 μM), respectively. This figure is representative of figures from three experiments.

Autophagy is generally considered as an important defense mechanism against aging and cellular senescence [8, 9]. It is thus paradoxical that HG-induced senescence is associated with enhanced autophagy. To unravel the paradoxical relationship, we treated LG-BMSC and HG-BMSC with 3-MA, an inhibitor of autophagy or rapamycin, an activator of autophagy and analyzed senescence. 3-MA did not exert a significant effect on LC3-II or MDC-positive autophagosomes in LG-BMSC, while rapamycin increased LC3-II and autophagosome formation in MSC cultured in LG (Figs 2C and 3). By contrast, 3-MA significantly reduced HG-induced LC3-II and autophagosomes while rapamycin induced only a moderate increase in LC3-II and autophagosome formation (Figs 2C and 3). We concurrently evaluated the effect of 3-MA and rapamycin on p21 expression and caspase 3 activation. Autophagy inhibition by 3-MA did not significantly alter p21 or caspase 3 in LG-BMSC but resulted in reduction of p21 and increase in caspase 3 in HG-BMSC (Fig 3). Activation of autophagy with rapamycin, on the other hand, had a minimal effect on p21 or caspase 3 in HG-BMSC but was associated with a significant reduction of caspase 3 (Fig 3). These results suggest that HG-induced autophagy elicits BMSC cell fate changes towards senescence and away from apoptosis. To support this, we determined additional cellular markers of senescence. 3-MA reduced SA-βgal positive cells (Fig 4A) increased cell proliferation (Fig 4B) and suppressed IL-6 production (Fig 4C). To confirm that 3-MA increases BMSC apoptosis, we analyzed cleaved PARP and measured TUNEL positive cells. 3-MA increased PARP cleavage (Fig 5A) and TUNEL-positive signals in HG-BMSC (Fig 5B) while rapamycin did not alter apoptosis. Taken together, these results suggest that HG-induced autophagy drives BMSC senescence but inhibits apoptosis. Further activation of autophagy with rapamycin does not exaggerate senescence.

**Fig 3:** HG-induced autophagy promotes senescence. BMSCs in LG or HG were treated with rapamycin, 3-MA or DMSO control for 48h. LC3-II, p21 and cleaved caspase 3 were analyzed by Western blotting. Upper panel shows representative blots and the low panel densitometry of Western blots. Error bars indicate mean ± SEM (n = 3). NS denotes statistically non-significant.

**Fig 4:** HG-induced autophagy promotes senescence and IL-6 released. **(A)** Analysis of SA-β-Gal by immunochemistry staining. Left panel shows representative figures and right panel, quantitative analysis of SA-β-Gal positive BMSCs. Error bars indicate mean ± SEM (n = 3). **(B)** BrdU incorporation was measured in BMSCs incubated with HG or LG for 28 days with or without rapamycin or 3-MA. **(C)** Measurement of IL-6 released into the medium by ELISA. Error bars refer to mean ± SEM (n = 3).

**Fig 5:** Suppression of HG-induced autophagy increases BMSC apoptosis. **(A)** Cell apoptosis was analyzed by cleaved PARP (cPARP) and **(B)** TUNEL positive signals. BMSCs in LG or HG were treated with rapamycin (RA), 3-MA or DMSO control for 48h. Error bars refer to mean ± SEM (n = 3).

### Antioxidants block HG-induced autophagy and senescence

Reactive oxygen species (ROS) were increased in BMSC cultured in HG as compared to that in LG (Fig 6A). However, ROS signals in HG-BMSC were approximately half of those generated by H_2_O_2_ treatment. To determine whether ROS are involved in BMSC autophagy and senescence, we pretreated BMSC with NAC before subjecting them to HG. NAC prevented HG-induced upregulation of Beclin-1 as well as Atg 5, 7 and 12 (Fig 6B) and blocked HG-induced autophagosome formation (Fig 6C). NAC abrogated HG-induced LC3-II which is accompanied by reduction of p21 protein levels (Fig 7A). Furthermore, NAC increased BrdU incorporation (Fig 7B), blunted HG-induced SA-βgal positive cells (Fig 7C) and suppressed IL-6 (Fig 7D). DPI, a NADPH oxidase inhibitor, blocked Atg expression (Fig 6B), and autophagosome formation (Fig 6C) and LC3-II generation (Fig 7A) to an extent comparable to NAC. Furthermore, DPI blocked HG-induced p21, increased BrdU incorporation, inhibited SA-βgal and suppressed IL-6 (Fig 7A–7D) in a manner comparable to NAC. Neither NAC nor DPI influenced TUNEL signals or cleaved PARP while H_2_O_2_ increased both (Fig 8A and 8B). These results suggest that HG-induced autophagy and senescence are mediated by ROS while control of apoptosis by HG is independent of ROS.

**Fig 6:** Antioxidants abrogate HG-induced autophagy. **(A)** The levels of ROS were measured by DCFH assay. H_2_O_2_ (750μM) was included as a positive control. **(B)** BMSCs in LG or HG were treated with NAC (5 mM) DPI (5 μM) or DMSO control for 48h. Beclin-1, Atg 5, 7 and 12 transcripts were analyzed by qPCR. The error bars indicate mean ± SEM (n = 3). **(C)** Analysis of autophagy by MDC staining.

**Fig 7:** Antioxidants suppress HG-induced senescence and IL-6 production. **(A)** LC3 and p21 were analyzed by Western blotting. Upper panel shows representative blots and the lower panel, densitometric analysis of blots. Error bars denote mean ± SEM (n = 3). NS denotes statistically non-significant. **(B)** BrdU incorporation was measured in BMSCs incubated with HG or LG for 28 days with or without NAC or DPI. **(C)** Upper panel shows representative figures of SA-β-Gal staining. The low panel, SA-β-Gal positive cells. Error bars denote mean ± SEM (n = 3)). **(D)** Measurement of IL-6 in the medium by ELISA. Error bars indicate mean ± SEM (n = 3). NS denotes statistically non-significant.

**Fig 8:** Neither NAC nor DPI influences BMSC apoptosis. **(A)** Cell apoptosis was analyzed by cleaved PARP and **(B)** TUNEL positive signals. BMSCs in LG or HG were treated with NAC, DPI or DMSO control for 48h. H_2_O_2_ (750μM) was included as a positive control. Error bars refer to mean ± SEM (n = 3).

## Discussion

In this study, we have shown that BMSC cultured in HG for 28 days display morphological changes and growth arrest, express p16, p21 and SA-βgal and secrete IL-6. These phenotypes are consistent with premature senescence. Cells cultured in LG for 28 days do not exhibit signs of senescence. It was reported that BMSCs cultured in LG do not start to display replicative senescent phenotype until they have been cultured for more than 43–77 days [10]. Our results indicate that HG induces BMSC senescence via upregulating autophagy. Antioxidants such as NAC and DPI block reactive oxygen species (ROS) thereby preventing autophagy and senescence. 3-MA prevents senescence by inhibiting autophagy. A schematic illustration of the pathway via which HG induces autophagy and senescence is shown in Fig 9.

**Fig 9:** Schematic illustration of the pathway via which HG induces autophagy and senescence. Antioxidants such as NAC blocks reactive oxygen species (ROS) thereby preventing autophagy and senescence. 3-MA prevents senescence by inhibiting autophagy.

Our data show that BMSCs are highly sensitive to the extracellular glucose concentrations (Fig 1). Most differentiated cells require HG in the culture medium for optimal growth. By contrast, BMSCs undergo premature senescence in HG environment. The reason for the differential handling of extracellular glucose is unclear. It has been suggested that extracellular glucose exerts its effect on cells not only through glucose metabolism, but also by metabolism-independent biochemical processes [11].

Autophagy is generally considered as an important defense mechanism against aging and cellular senescence [8, 9]. However, our data indicate that HG-induced senescence is associated with enhanced autophagy (Figs 2–4 and 7). Our findings provide an explanation for what appears to be conflicting reports regarding the influence of autophagy on cellular senescence. It was reported that deletion of autophagy-related genes accelerates cell senescence [12, 13] while oncogenic stresses induces senescence through activation of autophagy [14]. It is unclear why autophagy exerts opposite effects on cell senescence. A recent report suggests that stress-induced senescence is determined by the extent of autophagy [15]. It is possible that a “housekeeping” level of autophagy is required to prevent cellular senescence while excessive autophagic activation triggers senescence. HG induces excessive autophagy through upregulation of the expression of Atgs including Beclin-1. Autophagy was reported to control apoptosis through a crosstalk between Atg and caspase activation [16]. Our results reveal that HG-induced autophagy protects BMSCs from apoptosis. Thus, autophagy is pivotal in deciding the fate of BMSCs. When BMSCs are under HG stress, they turn up the autophagy machinery which switches on senescence and shuts down the apoptotic process. Autophagy-mediated senescence represents an important mechanism to keep BMSC alive. It is to be noted that even among differentiated cells, there is a variable response to HG stress. For example, renal podocytes in HG exhibit reduced autophagy which is accompanied by enhanced glomerular injury [17] whereas pancreatic β-cells in HG show increased autophagy which protects against cell death [18].

Senescent cells display senescence-associated secretory phenotype (SASP) with production of pro-inflammatory cytokines, proteases and growth factors [19]. SASP contributes to chronic inflammation in aging and is considered to be a major factor in the pathogenesis of age-related diseases [19]. As IL-6 is a key pro-inflammatory cytokine in SASP, we analyzed IL-6 release in HG-induced senescent BMSC and detected a four-fold increase in HG- vs. LG-BMSCs. Thus, HG-induced senescent BMSCs are kept alive through inhibition of apoptosis but acquire a secretory pro-inflammatory phenotype. Senescent BMSCs may play an important role in bone marrow niche dysfunction and hematopoietic impairment.

Several reports have shown that HG induces ROS generation which is responsible for cell damage and apoptosis [20, 21]. Little is known about ROS generation by HG in BMSCs nor is it known whether ROS induces senescence. In this study, we demonstrate that antioxidants such as NAC and DPI abrogate HG-induced autophagy and senescence (Figs 6–8). Since inhibition of NADPH oxidase by DPI exerts a comparable inhibition of HG-induced autophagy and senescence as NAC, HG probably induces ROS generation in BMSCs primarily through activation of NADPH oxidase. ROS was reported to trigger autophagy through Atg 4 cysteine oxidation [22]. Our results suggest that ROS activate autophagy by upregulating Atgs expressions.

Our findings have important therapeutic implications. BMSCs are key functional cell type that maintains hematopoietic niche. HG-induced BMSC senescence may cause cell reduction and hence alter niche function and impair hematopoiesis. Furthermore, HG-induced BMSC senescence releases pro-inflammatory cytokines which induce local inflammation and tissue damage. Since antioxidants are effective in preventing HG-induced BMSC senescence, NAC which was used in a large number of clinical trials for diverse human diseases [23, 24] may be valuable for treating hyperglycemia-induced niche dysfunction and hematopoietic defect.
